The article "Multifaceted Cerebral Venous Thrombosis With Extensive Intra-cerebral Hemorrhage in a Young Man With Mitral Valve Replacement Due to Thrombosis and IgA Nephropathy: A Challenging Case Report From Saudi Arabia" was published in 2024. Journal: Cureus.

# Multifaceted Cerebral Venous Thrombosis With Extensive Intra-cerebral Hemorrhage in a Young Man With Mitral Valve Replacement Due to Thrombosis and IgA Nephropathy: A Challenging Case Report From Saudi Arabia

**DOI:** 10.7759/cureus.60016

**Published:** 2024-05-10

**Authors:** Bashaier G AlQahtani, Naim Kajtazi, Hanan K Aljaidi

**Affiliations:** 1 Neurology, Prince Sultan Military Medical City, Riyadh, SAU

**Keywords:** young adult male, saudi arabia, antiphospholipid antibody syndrome, intracerebral hemorrhage, cerebral venous thrombosis

## Abstract

Cerebral venous thrombosis (CVT) is a cerebrovascular condition characterized by cerebral venous sinus thrombosis, resulting in venous infarction. The condition can manifest through a range of signs and symptoms such as headaches, benign intracranial hypertension, subarachnoid hemorrhage, localized neurological deficits, seizures, unexplained changes in consciousness, and meningoencephalitis. Its causes are linked to numerous different conditions and factors. We report a complicated case and course of antiphospholipid antibody syndrome in a young patient.

The case began two years prior, involving a 33-year-old man who had chronic kidney disease due to IgA nephropathy, pneumonia, and a large mass on his native mitral valve. He developed deep vein thrombosis (DVT) in his upper limb, for which he was prescribed warfarin. He was transferred to our hospital with a five-day history of severe headaches followed by a decrease in consciousness and seizures requiring intubation. He was found to have a subdural hematoma with a high international normalized ratio (INR). He underwent hematoma evacuation and a right decompressive craniotomy. CT of the brain via CT venography revealed intracerebral haemorrhage along with ischemic infarction in the right frontal-parietal and temporal lobes and cerebral venous thrombosis. He was treated with heparin infusion but later developed heparin-induced thrombocytopenia (HIT) and was switched to fondaparinux. Plasma exchange and intravenous methylprednisolone were given. His hospital course was complicated by recurrent infections, a new left intraparenchymal hemorrhage with intraventricular extension, and the need for extra ventricular drainage (EVD). The diagnosis of antiphospholipid antibody syndrome was confirmed.

This case report provides invaluable insights into managing a complex scenario that requires balanced decisions between anticoagulation in the context of severe ICH and the necessity of immunosuppressive therapy. The emphasis is on the significance of using a personalized and multidisciplinary strategy to address CVT situations and their issues.

## Introduction

Cerebral venous thrombosis (CVT), which involves thrombosis of the cerebral veins and dural sinuses, is a rare condition with an estimated annual incidence of three to four cases per million [1]. CVT can present with diverse signs and symptoms, including headache, benign intracranial hypertension, subarachnoid hemorrhage, focal neurological impairment, seizures, unexplained altered sensorium, and meningoencephalitis [2]. CVT can be caused by thrombophilia, oral contraception, infection, head and neck trauma, or neck surgery [3]. Despite recent breakthroughs in the detection of CVT, diagnosis and therapy may be difficult because of the wide range of underlying risk factors [4]. An uncommon case of intracerebral hemorrhage (ICH) caused by CVT in a young man who underwent mitral valve replacement due to thrombosis and IgA nephropathy is described.

The article "Multifaceted Cerebral Venous Thrombosis With Extensive Intra-cerebral Hemorrhage in a Young Man With Mitral Valve Replacement Due to Thrombosis and IgA Nephropathy: A Challenging Case Report From Saudi Arabia" was published in 2024. Journal: Cureus.

## Case presentation

A 33-year-old man without chronic disease was fine until the post-corona vaccine (about three years ago) when he developed acute febrile illness with denigrated renal functions, and renal biopsy showed IgA nephropathy. He was started on steroids, which led to an improvement in his condition. One and a half years ago, he developed hemoptysis and was found to have a large mass on the native mitral valve (tumor versus a thrombus or vegetation) and required metallic valve replacement (His cardiac condition, which necessitated a metallic valve replacement, was previously reported in the literature [5]). The patient has a medical history of deep vein thrombosis (DVT) in the upper limb, for which he was prescribed warfarin.

He was off immunotherapy for unknown reasons. On December 28, 2023, the patient arrived at our hospital unconscious with a history of severe headaches for five days before losing consciousness, which led to his admission. A subdural hematoma with a high international normalized ratio (INR) level was discovered. In addition, he had the onset of convulsions and subsequently required intubation. Anticoagulant medication was halted after the CT scan of the brain revealed a subdural hematoma (SDH) with radiological features of ischemic infarction affecting the right frontal-parietal and temporal lobes, as well as cerebral venous thrombosis. Also, the patient's father reported noticing mouth ulcers. Additional historical information showed that one of the patient's sisters had passed away at a young age due to issues related to systemic lupus erythematous. The initial CT scan revealed several hemorrhages, hypodensities, and a significant mass effect on the right side of the brain. The patient experienced anisocoria and endured a significant right craniotomy (Figure 1). The neurosurgeon observed thrombosed veins during the surgery. A magnetic resonance imaging (MRI) (Figure 2), magnetic resonance angiography (MRA), and magnetic resonance venography (MRV) brain scan revealed bilateral acute infarcts with bleeding, indicating venous infarction with SSS (superior sagittal sinus) thrombosis. The patient was initiated on heparin infusion according to the CVT protocol. The drug acetazolamide was administered. It was decided to start him on plasma exchange and IV methylprednisolone for three days, followed by IV hydrocortisone, for probable systemic vasculitis after consulting the hematology and rheumatology teams and to consider a stronger line of immunosuppressant agents whenever his general condition and infections improve. He underwent only three sessions of plasma exchange due to his ongoing problem with recurring infections, specifically upper respiratory tract infections (URTI) and urinary tract infections (UTI). The infusion of heparin was changed to fondaparinux because the patient had been diagnosed with heparin-induced thrombocytopenia (HIT) linked to cerebral venous thrombosis. No clinical seizures were observed, and the most recent electroencephalogram (EEG) indicates an encephalopathic pattern. The antiepileptic medication valproate was replaced with levetiracetam.

The article "Multifaceted Cerebral Venous Thrombosis With Extensive Intra-cerebral Hemorrhage in a Young Man With Mitral Valve Replacement Due to Thrombosis and IgA Nephropathy: A Challenging Case Report From Saudi Arabia" was published in 2024. Journal: Cureus.

**Figure 1:** Complex vascular abnormalities in brain CT scan, suggestive of venous thrombosis, presenting with multiple subdural and intracerebral hematomas in the right frontal and left parietal lobes.

**Figure 2:** Significant ischemic infarction in the right hemisphere with hemorrhage and mineralization on MRI.

The patient was referred to the cardiology department due to concern about cardioembolic causes. An echocardiogram (ECG) showed an ejection fraction (EF) of 55%. The mitral valve prosthesis was found to be intact, with no paravalvular leak or thrombus. The patient was advised by the nephrology team and received regular hemodialysis treatment (CRRT). He was confirmed to have antiphospholipid antibody syndrome. Significant clinical progress was observed, and the patient was successfully extubated following the insertion of a tracheostomy tube. However, during the hospital course developed a new left parieto-occipital hemorrhage with intraventricular extension that required EVD (extra ventricular drainage) insertion. He occasionally needs a small quantity of sedation to manage his anger. However, when not under sedation, he can open his eyes and respond to basic instructions.

## Discussion

Cerebral venous thrombosis (CVT) is a neurological disorder characterized by the blocking of cerebral veins, leading to venous infarction and intracerebral hemorrhage (ICH). A comprehensive review involving 8,829 individuals with CVT across 74 studies revealed an average patient age of 32.9 years, with females comprising 64.7% of the cases [6]. Our patient was within the reported average age range.

The article "Multifaceted Cerebral Venous Thrombosis With Extensive Intra-cerebral Hemorrhage in a Young Man With Mitral Valve Replacement Due to Thrombosis and IgA Nephropathy: A Challenging Case Report From Saudi Arabia" was published in 2024. Journal: Cureus.

Clinically, the sequence of headaches, followed by diminished consciousness and seizures, as exhibited by our patient, is commonly observed and necessitates immediate medical attention [7].

The diagnosis of CVT was confirmed by detecting thrombosis in the cerebral veins or sinuses, utilizing one of three imaging modalities: MRI with MR venography, CT with CT venography, or angiography. MRI is preferred for its superior sensitivity in identifying CVT across all thrombosis stages, with MR venography being particularly recommended for suspected cases of CVT. It has been noted that approximately 30% to 40% of CVT cases manifest with ICH [6].

According to the literature, for the treatment of CVT patients, initial anticoagulation with adjusted-dose unfractionated heparin or weight-based low-molecular-weight heparin in total anticoagulant dosages is appropriate, followed by vitamin K antagonists, regardless of ICH [3].

Ferro et al. developed and validated a risk score model to predict poor outcomes following CVT. The risk score model ranged from 0 (lowest risk) to 9 (highest risk), with a 3-point cut-off indicating a greater chance of mortality or dependency after six months. Malignancy, coma, or deep venous thrombosis was allocated two points each, while male sex, decreased degree of consciousness, or ICH received one point [8]. In the present case, male gender, a decreased degree of consciousness, deep venous thrombosis, and ICH were detected. Hence, this case scored 5 points and was classified as severe. Although the patient in the present study was in the high-risk group, early detection and treatment resulted in a favorable outcome. Careful follow-up is required because 4.4% of CVT patients experience recurrence [9].

## Conclusions

The major takeaway from the case report emphasizes the importance of a personalized and multidisciplinary approach to managing cerebral venous thrombosis (CVT) and its complications. This involves maintaining a high level of suspicion for CVT, especially in patients presenting with non-specific symptoms such as headaches, altered consciousness, and seizures. Comprehensive diagnostic evaluations, including neuroimaging and laboratory tests, are crucial for facilitating early intervention.
